This article has been retracted.

# Effects of Continuous Care Combined with Evidence-Based Nursing on Mental Status and Quality of Life and Self-Care Ability in Patients with Liver from Breast Cancer: A Single-Center Randomized Controlled Study

**DOI:** 10.1155/2022/3637792

**Published:** 2022-04-28

**Authors:** Xin Zhang, Di Zhang, Peidan Yu, Xuemei Li

**Affiliations:** Hubei Cancer Hospital Breast Department, 43000, China

## Abstract

**Objective:**

To explore the multidisciplinary collaborative extended care combined with EBN to improve breast cancer liver metastasis patients' psychological status and self-care ability.

**Background:**

In the past ten years, the number of breast cancer patients with liver metastases has increased year by year, becoming a global public health problem. Studies have shown that 30% of breast cancer patients with liver metastases show varying degrees of anxiety and depression, and their quality of life is significantly lower than that of the normal population. Multidisciplinary collaborative continuous care can improve the prognosis of breast cancer treatment to a certain extent and is the key to meeting the needs of cancer patients.

**Materials and Methods:**

The clinical data of 96 patients with liver metastases from breast cancer were selected as the study subjects and divided into a comparison group and an observation group of 48 cases each according to a random number table. Among them, the comparison group implemented evidence-based nursing (EBN) and the observation group implemented multidisciplinary collaborative extended care based on the comparison group. The effects of psychological status, quality of life, self-care ability, and sleep quality were compared between the two groups before and after nursing care.

**Results:**

After nursing, the sleep quality scores, increased awakening scores, sleep quality that shows weakness because important things are not steady or strong scores, and night terrors scores of the two groups of breast cancer patients with liver the spread of diseases through the body were very much improved, and the sleep quality scores of the instance of watching, noticing, or making a statement group were much lower than those of the comparison group (*P* < 0.05). After nursing, the fear and stress-related score, depression score, tiredness and distress score, and anger score of the two groups of breast cancer patients with liver (the spread of diseases through the body) were very much improved, and the mental state score of the instance of watching, noticing, or making a statement group was much lower than that of the comparison group (*P* < 0.05). The scores of self-care skills, self-responsibility, health knowledge, and self-idea of patients in the instance of watching, noticing, or making a statement group after nursing were higher than those in the comparison group (*P* < 0.05). After nursing, the scores of mental energy, social interaction, emotional restriction, and mental status of patients in (instance of watching, noticing, or making a statement) were much higher than those in the comparison group (*P* < 0.05).

**Conclusion:**

Multidisciplinary collaborative continuous nursing combined with EBN can effectively improve the sleep quality and psychological state of patients with breast cancer and liver metastases and improve self-care ability.

## 1. Introduction

Breast cancer is the most common female malignant tumor, and its incidence is increasing year by year. It has been reported in the literature that nearly 1/3 of breast cancer patients will develop to an advanced stage, and the prognosis of advanced breast cancer is poor, with a five-year survival rate of about 20% [1]. Liver metastasis of breast cancer is a common metastatic site of advanced breast cancer, and some foreign reports show that the incidence of liver metastasis from breast cancer is greater than 50% [2]. However, the incidence of isolated liver metastases as the first metastases is relatively low. The liver is a vital internal organ. Once the metastasis occurs in this site, the prognosis is poor, and it is reported in the literature that liver metastasis from breast cancer can only survive for up to 20 months [3]. Once liver metastases from breast cancer occur, most of them are multiple metastases accompanied by metastases in other sites, and only a few have the opportunity for local treatment [4]. However, the liver is an important “detoxification” organ of the human body. Most drugs need to be metabolized in the liver. After liver metastases occur, the function of the liver can be affected. The treatment of liver metastases from breast cancer is relatively difficult [5]. Liver metastasis of breast cancer will not only lead to physiological abnormalities in patients but also cause changes in female body shape due to surgery, leading to widespread anxiety, depression, and other negative emotions in patients, thereby affecting the patient's self-care ability and quality of life, which is not conducive to the recovery of prognosis [6].

Studies have found that multidisciplinary collaborative continuous nursing can improve the prognosis of breast cancer liver metastases to a certain extent [7]. Multidisciplinary collaborative continuous nursing can enable patients to obtain scientific and continuous rehabilitation guidance in different places such as hospitals and families, which is of positive significance for satisfying the care of patients after discharge and can promote the early recovery of patients and reduce the rate of rehospitalization [8]. Using different kinds of expert knowledge (group/working well together), continuous nursing has been established earlier in foreign countries and has developed more maturely. Especially in developed countries, patients have done an excellent job of changing (from one thing to another) between different nursing opportunities. With the increase of patient care needs (using different kinds of expert knowledge group), continuous nursing has become a popular thing (the general way things are going) of medicine-based nursing [9]. Therefore, based on medicine-based treatment, this study compared the application effect of EBN and using different kinds of expert knowledge groups working well together continuous nursing on the nursing of patients with liver the spread of diseases through the body from breast cancer. Therefore, this study explores the influence of using different kinds of expert knowledge group together continuous nursing on the mental state, quality of life, self-care ability, and sleep quality of patients with liver (the spread of diseases through the body from breast cancer) and provides a reference basis for medicine-based nursing of patients with liver (the spread of diseases through the body) from breast cancer. The report is as follows.

## 2. Material and Methods

### 2.1. Research Object

The medicine-based data of 96 patients with liver the spread of diseases through the body from breast cancer who were treated in our hospital from August 2018 to August 2021 were selected as the research objects, and they were divided into comparison groups and instances of watching, noticing, or making a statement group with 48 cases each according to the random number table. Comparison group: old/allowed to get old/got older 45-75 years, mean (67.4 ± 13.7) years old; 20 patients with first or most crucial tumor stage I-II, 28 patients with stage III-IV, of which 6 patients had the distant disease when they were found spreading of disease; education level: 3 cases of inability to read and write, 10 cases of junior high school education, 12 cases of high school education, and 23 cases of college education or above; an instance of watching, noticing, or making a statement group: age 47-81 years old, average (61.9 ± 13.8) years old; first or most important tumor stage is I-II. There were 23 patients with stage III-IV and 25 patients with stage III-IV, of which 8 patients had distant the spread of diseases through the body when they were found; education level: 4 were unable to read and write, 12 had junior high school education, 10 had high school education, and 22 had a college education. The general data of the two groups of patients are similar; *P* > 0.05, not related to studying number difference, which can be compared.

### 2.2. Inclusion and Exclusion Criteria

Inclusion criteria are as follows: (i) the selected patients with liver metastases from breast cancer met the diagnostic criteria of the “China Consensus Guidelines for Advanced Breast Cancer (CABC 2015)” [10] and were histopathologically diagnosed with breast cancer; (ii) had breast cancer diagnosed by imaging (including B-ultrasound, CT, PET-CT, or MRI) or pathologically confirmed intrahepatic metastases, and the largest diameter of the metastases is greater than or equal to 1 cm; and (iii) the patient can surf the Internet and use a smartphone, is conscious, has normal intelligence, and has good Chinese comprehension ability.

Exclusion criteria are as follows: (i) patients with other cancers, or breast cancer metastasized from other cancers, and patients with severe heart, liver, and kidney dysfunction; (ii) patients with severe mental disorders, severe endocrine dysfunction or blood system diseases, poor compliance, and unable to cooperate with investigators; and (iii) patients with coagulation disorders, pregnant and lactating women, those with a survival period of less than 1 year, and those with expression disorders or mental illness.

### 2.3. Nursing Intervention Methods

#### 2.3.1. EBN

The comparison group implements EBN, that is, according to the comprehensive and accurate assessment of nursing problems, the selection of optimal methods, and the formulation and implementation of nursing interventions. First of all, a comprehensive evaluation and systematic analysis of the patient's disease itself, complications of the surgery, radiotherapy and chemotherapy, psychological, emotional, and family environment are collected from nursing observations. Carry out a relevant literature search for existing and potential nursing problems of patients, find the best method from the network system of the hospital information department and journals, etc., look for scientific and reasonable evidence, and combine the actual situation of the patient to formulate effective nursing and preventive measures.

- Psychological factors play a vital role in cancer occurrence, development, and prognosis [2]. Among various diseases, few such as cancer give people great mental pressure and produce bad psychological emotions. Due to the long course of radiotherapy and chemotherapy after breast cancer surgery, patients have different degrees of anxiety, depression, fear and anger, and other negative emotions, affecting the patient's treatment and quality of life. Therefore, good psychological care of patients is an important part of completing treatment and improving the quality of life of patients. Nurses need to find relevant knowledge of psychology, conduct psychological counseling according to the different cultural qualities, personality characteristics, and psychological states of patients, and implement targeted personalized nursing. Operation, targeted retrieval of relevant theoretical knowledge, such as the special treatment of tumor patients, examination methods and the role of drugs, side effects and treatment prospects, etc., timely answer questions, eliminate patients' doubts, and tell patients that as long as they adhere to regular treatment. Normal people live and work the same way, actively mobilize the patient's inherent ability to cope with crises, strengthen the patient's will to fight cancer, maintain emotional stability, face cancer with an optimistic attitude, and receive treatment
- Postoperative radiotherapy and chemotherapy can kill tumor cells and damage normal tissue cells to varying degrees. Strengthening nutrition plays an important role in promoting tissue repair, improving treatment effects, and reducing toxic and side effects. In addition, tumor chemotherapy patients often have nausea, vomiting, diarrhea, resulting in loss of water and nutrients, and emotional depression makes patients lack appetite. Reasonable nutritional support can correct the malnutrition of tumor patients, improve nutritional status, and enable patients to tolerate better. Chemotherapy is to boost immunity. It is necessary to strengthen the education of patients and their families about nutritional diet knowledge, pay attention to the scientific and reasonable combination of diets, and take high-protein, high-vitamin, high-calorie, light, and easily digestible diets as the standard. If the white blood cells decrease during radiotherapy and chemotherapy, instruct the patient to eat some foods rich in nutrients, such as jujube porridge, turtle meat, pig stomach soup, astragalus, and black chicken soup
- The skin elasticity of breast cancer patients is poor after surgery, especially the skin tissue in the radiotherapy area is thin, which is prone to skin reactions. The patient should be assisted in personal hygiene, and the patient should be told to wear cotton underwear to avoid friction and pressure on the skin in the radiotherapy area. Use harsh detergents, etc. Through a literature search, it is also known that aloe vera has good antiulcer and anti-inflammatory effects, covering the surface of ulcers and inflammation, which can protect the mucosa and promote cell regeneration

### 2.4. Multidisciplinary Collaborative Continued Care

The observation group implements multidisciplinary collaborative continuous nursing based on the comparison group, that is, (1) establishes a multidisciplinary collaborative continuous nursing team, which consists of a head nurse, 2 nurses specialized in oncology, a breast doctor, a psychologist, and 1 nutritionist. (1) Specialist nurses are mainly responsible for explaining disease-related knowledge and instructing patients on self-care guidance. (2) Breast physicians are mainly responsible for comprehensively evaluating the patient's general condition and treatment effect, explaining breast cancer-related knowledge, drug dosage, and treatment of adverse reactions. (3) The psychologist is mainly responsible for the psychological sorting out of the patient, communicates with the patient in gentle words, understands the inner thoughts of the patient, and uses professional and scientific methods to sort out the psychological problems of the patient. (2) 3 days before discharge, the multidisciplinary collaborative continuous nursing team will conduct a comprehensive assessment of the patient and formulate a corresponding individualized continuous nursing plan; establish a nursing team and a patient communication group, and patients can leave a message in the group at any time to communicate with medical staff. After discharge, return to the patient once a week to fully understand the implementation of continuous nursing care, actively answer the patient's questions during this period, and communicate with the patient and their family members to adjust the nursing plan; 3 months after discharge, go back to the hospital for a review. The intervention period was from before intervention to 3 months after discharge.

### 2.5. Observation Indicators

(1) Sleep status self-rating scale evaluates the sleep quality of patients, including four items: sleep quality, increased awakening, sleep instability, and night terrors. Each item is scored from 0 to 5. (2) The psychological state score was evaluated according to the Brief Mood Scale (BPOMS), including four items of anxiety, depression, fatigue and distress, and anger, with a score of 0-7 for each item. The higher the score, the greater the emotional response. (3) Self-care ability score: the self-care ability score of the two groups was compared using the self-care ability measurement scale before the action that helps a bad situation and 3 months after the action that helps a bad situation, including 4 items: self-care skills, health knowledge, self-idea, and self-responsibility. There are 43 items, each item has a score of 0-4 points, and the total score is 172 points. The higher the score, the stronger the patient's self-care ability. (4) Quality of life score: it includes four parts: mental energy score, social interaction score, emotional limitation score, and mental status score, each of which is scored from 0 to 100. The higher the score, the better the quality of life of patients with liver the spread of diseases through the body from breast cancer. The Cronbach's alpha values of the above scales were all greater than 0.914 before use. Breast cancer patients with liver spread diseases through the body filled in independently without being affected by any internal and external factors.

### 2.6. Statistical Analysis

All data for this study were entered in full using Epidata, and then, SPSS 25.0 was used to statistically process the data. The data needs to be entered into a computer database by a second person to ensure the completeness and accuracy of the data. *χ*^2^ test is used to express the count data as a percentage (%). For each parameter, data is mentioned as mean ± SD and statistically analyzed by employing one-way ANOVA followed Tukey's multiple comparisons post hoc test. *P* < 0.05 is considered statistically significant.

## 3. Results

### 3.1. Sleep Quality Score Comparison

After nursing, the sleep quality scores, increased awakening scores, sleep instability scores, and night terrors scores of breast cancer patients with liver metastases in the two groups were significantly improved. The sleep quality scores of the observation group were significantly lower than those of the comparison group. There was statistical significance (*P* < 0.05) (see Figure 1).

### 3.2. Mental State Comparison

After nursing, the anxiety score, depression score, fatigue and distress score, and anger score of the two groups of breast cancer patients with liver metastases were significantly improved, and the psychological state score of the observation group was significantly lower than that of the comparison group, and statistics showed that the difference was statistically significant (*P* < 0.05) (see Figure 2).

### 3.3. Self-Care Ability Score Comparison

There was no statistically significant difference in the self-care ability scores between the two groups before care (*P* > 0.05). At the end of care, the observation group had higher self-care, self-responsibility, health knowledge, and self-concept scores than the control group. In statistics, this difference proved to be statistically significant (*P* < 0.05) (see Figure 3).

### 3.4. Quality of Life Score Comparison

After nursing, the scores of mental vitality, social interaction, emotional limitation, and mental status of the observation group were significantly higher than those of the comparison group, and the difference was statistically significant (*P* < 0.05) (see Figure 4).

## 4. Discussion

Breast cancer is a serious disease affecting women's health, the cause of which is not fully understood and is generally thought-about to be related to the timing of first menstrual period and menopause, radiation, mental factors, and other sicknesses [11]. Now, involving surgery that removes a lot of diseased tissue, bone, etc., is the main treatment for breast cancer. However, most patients are influenced by factors such as the study of beauty and pain after an operation, and their obedience to functional exercise is less than ideal, which reduces prediction-related results and quality of life [12]. EBN is taken from medical events or objects that prove something, which refers to the process of nursing staff combining scientific findings with medicine-based experience and patient wishes in the planning of nursing activities to prove something as a basis for medicine-based nursing the process of making decisions based on it [13–15]. Nursing staff search for and identify problems in medicine-based practice, specify and structure them, and conduct a well-thought-out search of the clearly connected or related books based on the questions presented asked stood in a showy way to find external evidence that was seen coming from the research [16]. The scientific events or objects prove something was reviewed for something is truly what it claims to be and ability to be applied to broader situations. The reviewed scientific events or objects that prove something was combined with medicine-based knowledge and experience and patient needs, and a care plan based on the medical information that proves something was made to meet the patient's needs [17, 18]. The care plan is used, and the effectiveness of the (putting into use) medical information that proves something is supervised through self-test, fact-checking and careful reading by other educated people doing the same work, and approval from an organization [19]. Therefore, we conducted an EBN measure for breast cancer patients, and thorough review, we found that reading and writing ability, mental status, related to vitamins, protein, etc. in food support, sicknesses that happen along with other sicknesses, and after-discharge care needs were all connected or related factors affecting the outlook of patient care [20]. However, EBN is unable to provide long-term extended care to patients with adverse conditions. Through the joint efforts of different types of specialists to improve the quality of life of patients with liver disease whose breast cancer has spread into the body, reduce mental state and improve the quality of sleep, in favor of patients with further medications or other treatments) [21].

In this study, both sleep and night terrors in liver patients have been greatly improved, and the use of different kinds of prolonged care combined with EBN can effectively improve sleep quality [22]. This may be due to the use of different types of care and corresponding care measures [23]. Poor sleep quality is that the patient is not satisfied with the sleep time or sleep quality, which affects its social functioning during the day, mainly manifested in sleep (sleep delay), early awakening (inability to fall asleep) may increase the patient's pain and heavy burden of money, and medical staff should take it seriously [24–26]. These main nursing measures are to determine the factors affecting patients' sleep by actively communicating with them, making mental recalculations and behavioural guidance, and encouraging patients to treat them correctly with a positive thinking and confident attitude [27]. Counsel patients to better adapt to the new environment, control unpleasant feelings such as love, hate and fear, respect and protect patients' privacy and self-confidence, and establish a pleasant nurse-patient relationship [28].

After the care in this study, the fear and stress-related score, depression score, tiredness sleepiness score, and anger score of breast cancer liver spreading of disease patients in both groups were very much improved, and the mental state score of the instance of watching, noticing, or making a statement group was much lower than that of the control group, pointing to/showing that using different kinds of working well together extended care combined with EBN can effectively improve the mental state of patients [29]. Breast cancer is different from other harmful tumors in that it brings physical pain and the effect on the physical form. Patients are likely to experience to get depression, shaking, and other bad feelings of love, hate, fear, etc., which seriously affect the recovery of the disease [30]. It is suggested that extended care based on using different kinds of expert knowledge working team effort has the effect of improving upset and depression in patients with liver the spread of diseases through the body from breast cancer.

In this study, the patients' self-care skills scores, self-responsibility scores, health knowledge scores, and self-concept scores were higher than those in the control group, indicating that using different types of expert knowledge group care combined with EBN can improve the patients' self-care ability. [31]. The clearly particular reasons for this are carefully studied as follows: self-care ability is the ability of an individual to maintain and improve the development of physical and mental health to go move forward and put into action, which is also a human gut feeling, and higher self-care ability is helpful to the health and well-being of a person's life [32–35]. Using different kinds of working well together extended care is the result of deliberately planning and trying something and planned nursing activity that gives a reason to do something patients to consciously hug/support healthful knowledge and develop healthy behaviors and way of living changes/recalculations, which in turn helps disease recovery [36]. Focus on continuous and constant care and follow-up after treatment [37]. At the same time, targeted education according to the patient's level of understanding has effectively improved the patient's knowledge rate and guided the patient's outlook in the follow-up work, helping the patient to develop good habits and improve their treatment confidence, this way helping increase in a good way disease recovery [38]. Modern nursing research shows that improving a patient's ability to self-care helps improve their ability to cope with the disease successfully and enables them to actively participate in the treatment of the disease, which can improve their condition [39].

The mental energy score, social interaction score, emotional limitation score, and mental status of patients in the instance of watching, noticing, or making a statement group were much higher than those in the control group aftercare in this study. It indicated that using different kinds of expert knowledge group extended care combined with EBN can effectively improve the quality of life of patients with liver the spread of diseases through the body from breast cancer. Analysis of its origin: EBN is a series of actions that help bad situations to make sure that patients remain well cared for after discharge from the hospital and is a continuation from hospital to home to help patients and their families improve their self-care skills [40]. Now, something commonly done care used in the clinic has slowly did not meet the needs of patients, and the out-of-hospital follow-up is more random and not in a way that is close to the truth or true number oriented to the actual condition of the patient. In contrast, using different types of cooperative care can help patients recover, can stimulate patients to participate in treatment actively, and can improve their quality of life through changes in thinking, thereby enabling a change in belief that makes the patient better.

This study has some invention of new things and some limits. First, the sample size of this study was small, and the selection of patients included to leave outpatients with liver the spread of diseases through the body from breast cancer was open to opinion and judging, not black-and-white due to different factors, such as age and reading and writing ability level, and most of the patients were old patients in areas away from cities with poor knowledge and low knowledge of the disease, so the results of the study may not be representative or created unfair thinking in. Second, using different kinds of working well together extended care has more limits in practice, such as lack of understanding of patients and their families, money-based conditions, uneven setting apart and distributing of medical useful things supplies, and many other factors that can affect patients' feelings of love, hate, fear, etc. This study did not conduct a complete and well-thought-out test/evaluation. Finally, the short length of time of the action that helps a bad situation and the uninterrupted, constant quality of care measures need to be further improved in the future. In the future, it is necessary to expand the sample size and extend the follow-up time to avoid adverse patient conditions.

## 5. Conclusion

Using different kinds of expert knowledge groups uninterrupted, constant quality of care combined with EBN can effectively improve the quality of life and mental status of patients with liver the spread of diseases through the body from breast cancer, improve self-care ability and sleep quality, which is helpful to patient outlook and medicine-based treatment, and provide a practical basis for accomplishing or gaining with effort hospital-family health management for other cancer patients in the future.

## Figures and Tables

**Figure 1:** Comparison of sleep quality scores (according to the test standard of *α* = 0.05, the scores of sleep quality (a), increased arousal score (b), sleep instability score (c), sleep disturbance scores of the two groups of breast cancer patients with liver metastases after nursing care, and night terrors scores (d) were significantly improved, and the sleep quality score in the instance of watching, noticing, or making a statement group was much lower than that in the comparison group. Values are expressed as mean ± SD and carefully studied by an independent sample *t*-test. After nursing, the instance of watching, noticing, or making a statement group's sleep quality score increased with a more excited or awake state than before, sleep quality shows weakness because important things are not steady or strong score, and night terrors score were lower than those of the comparison group (*P* < 0.05)).

**Figure 2:** Comparison of mental state scores (fear and stress scores (a), depression scores (b), tiredness and distress scores (c), and anger scores (d) were very much improved in both groups of breast cancer patients aftercare for liver (the spread of diseases through the body); (d) according to the $\hat{I}\pm =0.05$, test judging requirements and the mental state scores in the instance of watching, noticing, or making a statement group were much lower than those in the control group. Values are expressed as $\text{mean }\hat{A}\pm \text{standard}$ moving away and were analyzed by independent sample *t*-test. The fear and stress-related score, depression score, tiredness distress score, and anger score in the instance of watching, noticing, or making a statement group were lower than those in the control group aftercare (*P* < 0.05)).

**Figure 3:** Self-care ability score comparison (health knowledge score (c) and self-concept score (d) were significantly improved, and the observation group's self-care ability score was significantly higher than that of the comparison group. According to the test standard of *α* = 0.05, the values were expressed as mean ± SD which indicates that, using independent sample *t*-test analysis, the nursing skill score, self-responsibility score, health knowledge score, and self-concept score of the observation group after nursing were higher than those of the comparison group (*P* < 0.05)).

**Figure 4:** Comparison of quality of life scores (there was no big difference in the quality of life scores between the two groups before nursing (*P* > 0.05). After nursing, the scores of mental energy (a), social interaction (b), emotional restriction score (c), and mental status score (d) were very much improved, and the self-protection ability score of the instance of watching, noticing, or making a statement group was much higher than that of the comparison group. According to the test standard of $\hat{I}\pm =0.05$, the value was expressed as $\text{mean }\hat{A}\pm \text{SD}$, and the independent samples *t*-test was used for analysis. After nursing, the instance of watching, noticing, or making a statement group had higher scores of mental energy, social interaction, emotional limitation, and mental status than the comparison group (*P* < 0.05).

## Data Availability

No data were used to support this study.

## References

[1] Yousefi M., Nosrati R., Salmaninejad A., Dehghani S., Shahryari A., Saberi A. (2018). Organ-specific metastasis of breast cancer: molecular and cellular mechanisms underlying lung metastasis. *Cellular Oncology (Dordrecht)*.

[2] Pagani O., Senkus E., Wood W. (2010). International guidelines for management of metastatic breast cancer: can metastatic breast cancer be cured?. *Journal of the National Cancer Institute*.

[3] Wang R., Zhu Y., Liu X., Liao X., He J., Niu L. (2019). The clinicopathological features and survival outcomes of patients with different metastatic sites in stage IV breast cancer. *BMC Cancer*.

[4] Franzese C., Comito T., Viganò L. (2020). Liver metastases-directed therapy in the management of oligometastatic breast cancer. *Clinical Breast Cancer*.

[5] Arciero C. A., Guo Y., Jiang R. (2019). ER+/HER2+ breast cancer has different metastatic patterns and better survival than ER-/HER2+ breast cancer. *Clinical Breast Cancer*.

[6] Liang Y., Zhang H., Song X., Yang Q. (2020). Metastatic heterogeneity of breast cancer: molecular mechanism and potential therapeutic targets. *Seminars in Cancer Biology*.

[7] Reeves S., Pelone F., Harrison R., Goldman J., Zwarenstein M. (2000). Interprofessional collaboration to improve professional practice and healthcare outcomes. *Cochrane Database of Systematic Reviews*.

[8] Rovira A., Dawson D., Walker A. (2021). Tracheostomy care and decannulation during the COVID-19 pandemic. A multidisciplinary clinical practice guideline. *European Archives of Oto-Rhino-Laryngology*.

[9] Muth C., Blom J. W., Smith S. M. (2019). Evidence supporting the best clinical management of patients with multimorbidity and polypharmacy: a systematic guideline review and expert consensus. *Journal of Internal Medicine*.

[10] Professional Committee of Clinical Oncology of Chinese Women Physician Association, Professional Committee of Breast Cancer of China Anti-Cancer Association (2015). Consensus guidelines for advanced breast cancer in China (CABC 2015). *Cancer Progress*.

[11] Wu Q., Li J., Zhu S. (2017). Breast cancer subtypes predict the preferential site of distant metastases: a SEER based study. *Oncotarget*.

[12] Medeiros B., Allan A. L. (2019). Molecular mechanisms of breast cancer metastasis to the lung: clinical and experimental perspectives. *International Journal of Molecular Sciences*.

[13] Gooding D., Swift A. (2019). Use of social media to support student nurses: an EBN Twitter chat led by Daniel Gooding and Alison Twycross. *Evidence-Based Nursing*.

[14] Albishtue A. A., Yimer N., Zakaria M. Z. A. (2019). Effects of EBN on embryo implantation, plasma concentrations of reproductive hormones, and uterine expressions of genes of PCNA, steroids, growth factors and their receptors in rats. *Theriogenology*.

[15] Ma X., Zhang J., Liang J. (2019). Authentication of edible bird's nest (EBN) and its adulterants by integration of shotgun proteomics and scheduled multiple reaction monitoring (MRM) based on tandem mass spectrometry. *Food Research International*.

[16] Hun Lee T., Hau Lee C., Alia Azmi N. (2020). Characterization of polar and non-polar compounds of house edible bird's nest (EBN) from Johor, Malaysia. *Chemistry & Biodiversity*.

[17] Ling J. W. A., Chang L. S., Babji A. S., Lim S. J. (2020). Recovery of value-added glycopeptides from edible bird's nest (EBN) co-products: enzymatic hydrolysis, physicochemical characteristics and bioactivity. *Journal of the Science of Food and Agriculture*.

[18] Zwarenstein M., Goldman J., Reeves S. (2009). Interprofessional collaboration: effects of practice-based interventions on professional practice and healthcare outcomes. *Cochrane database of systematic reviews*.

[19] Connor M. J., Karakala N. (2017). Continuous renal replacement therapy: reviewing current best practice to provide high-quality extracorporeal therapy to critically ill patients. *Advances in Chronic Kidney Disease*.

[20] Patel H., Yirdaw E., Yu A. (2019). Improving early discharge using a team-based structure for discharge multidisciplinary rounds. *Professional Case Management*.

[21] Friesen L., Andersen E. (2019). Outcomes of collaborative and interdisciplinary palliative education for health care assistants: a qualitative metasummary. *Journal of Nursing Management*.

[22] Walton V., Hogden A., Long J. C., Johnson J. K., Greenfield D. (2019). How do interprofessional healthcare teams perceive the benefits and challenges of interdisciplinary Ward rounds. *Journal of Multidisciplinary Healthcare*.

[23] Kahn J. M., Kelly K. M. (2018). Adolescent and young adult Hodgkin lymphoma: raising the bar through collaborative science and multidisciplinary care. *Pediatric Blood & Cancer*.

[24] Castillo J., Castillo H., Thibadeau J. K., Brei T. (2021). Spina bifida care, education, and research: a multidisciplinary community in a global context. *Journal of Pediatric Rehabilitation Medicine*.

[25] Streiff M. B., Lau B. D., Hobson D. B. (2016). The Johns Hopkins venous thromboembolism collaborative: multidisciplinary team approach to achieve perfect prophylaxis. *Journal of Hospital Medicine*.

[26] Hsu H. T., Chiang Y. C., Lai Y. H., Lin L. Y., Hsieh H. F., Chen J. L. (2021). Effectiveness of multidisciplinary care for Chronic Kidney Disease: a systematic review. *Worldviews on Evidence-Based Nursing*.

[27] Fett N., Werth V. P. (2021). A multidisciplinary collaborative approach to retinal toxic effects screening for dermatology patients taking antimalarials. *JAMA Dermatology*.

[28] Zhao N., Yin F., Wu X., Zhong Y. (2020). The effectiveness of a WeChat-based multimodal nursing program for women with breast cancer: a randomized controlled trial protocol. *Medicine (Baltimore)*.

[29] Li H., Sun X., Miller E. (2017). BMI, reproductive factors, and breast cancer molecular subtypes: a case-control study and meta-analysis. *Journal of epidemiology*.

[30] Romieu I. I., Amadou A., Chajes V. (2017). The role of diet, physical activity, body fatness, and breastfeeding in breast cancer in young women: epidemiological evidence. *Revista de Investigación Clínica*.

[31] Corey B., Smania M. A., Spotts H., Andersen M. (2020). Young women with breast cancer: treatment, care, and nursing implications. *Clinical Journal of Oncology Nursing*.

[32] Johnson H. M., Mitchell K. B. (2019). Breastfeeding and breast cancer: managing lactation in survivors and women with a new diagnosis. *Annals of Surgical Oncology*.

[33] Tan M. M., Ho W. K., Yoon S. Y. (2018). A case-control study of breast cancer risk factors in 7,663 women in Malaysia. *PLoS One*.

[34] Sussman J., Bainbridge D., Whelan T. J. (2017). Evaluation of a specialized oncology nursing supportive care intervention in newly diagnosed breast and colorectal cancer patients following surgery: a cluster randomized trial. *Supportive Care in Cancer*.

[35] Carmichael H., Matsen C., Freer P. (2017). Breast cancer screening of pregnant and breastfeeding women with BRCA mutations. *Breast Cancer Research and Treatment*.

[36] Reinbolt R. E., Mangini N., Hill J. L. (2015). Endocrine therapy in breast cancer: the neoadjuvant, adjuvant, and metastatic approach. *Seminars in Oncology Nursing*.

[37] Zhou Y., Chen J., Li Q., Huang W., Lan H., Jiang H. (2015). Association between breastfeeding and breast cancer risk: evidence from a meta-analysis. *Breastfeeding medicine*.

[38] Unar-Munguía M., Torres-Mejía G., Colchero M. A., González de Cosío T. (2017). Breastfeeding mode and risk of breast cancer: a dose-response meta-analysis. *Journal of Human Lactation*.

[39] Wang X., Lai Q., Tian Y., Zou L. (2020). Effect of evidence-based nursing intervention on upper limb function in postoperative radiotherapy patients with breast cancer. *Medicine (Baltimore)*.

[40] Vila C., Reñones C., Ferro T. (2017). Advanced breast cancer clinical nursing curriculum: review and recommendations. *Clinical & Translational Oncology*.

